The article "Improved Watershed Algorithm-Based Microscopic Images Combined with Meibomian Gland Microprobe in the Treatment of Demodectic Blepharitis" was published in 2022. Journal: Comput Math Methods Med.

# Improved Watershed Algorithm-Based Microscopic Images Combined with Meibomian Gland Microprobe in the Treatment of Demodectic Blepharitis

**DOI:** 10.1155/2022/4389659

**Published:** 2022-06-08

**Authors:** Lanying Liu, Shengfu Yang, Min Zhu, Min Wang, Xin Wei

**Affiliations:** Department of Ophthalmology, 302 Hospital of China Guizhou Aviation Industry Group, Anshun City, Guizhou Province 561000, China

## Abstract

The objective of the study was to explore microscopic images under a watershed segmentation algorithm combined with meibomian gland microprobe in the treatment of demodectic blepharitis. For segmenting the connected target objects in the image, the watershed algorithm was utilized first to obtain the target region in the image, and then, the fuzzy *C*-means (FCM) clustering algorithm was used to cluster the targets. The different grayscale regions in the microscopic images were segmented. 90 patients with demodectic blepharitis-related dry eyes were selected, and they were divided into experimental group 1 (group E1, *n* = 30), experimental group 2 (group E2, *n* = 30), and control group (group CG, *n* = 30). The breakup time (BUT) of the tear film, the subjective score of clinical symptoms, and the number of mites were compared among the three groups before and after treatment. The results showed that after treatment, the indicators of group E1 and group E2 were significantly lower than those before treatment, and the differences were statistically significant (*P* < 0.05). The treatment effect of group E1 was significantly better than that of the other two groups (*P* < 0.05). The subjective clinical symptom scores of groups E1, E2, and CG were 13.43 ± 1.41, 13.51 ± 1.41, and 13.64 ± 0.84, respectively, before treatment, and those after treatment were 3.1 ± 1.841, 5.4 ± 0.661, and 13.4 ± 0.841, respectively. The clinical sign scores of the groups E1 and E2 after treatment were remarkably different from those before treatment (*P* < 0.05). Compared with the scores of clinical signs and clinical symptoms after treatment, those of group E1 showed the largest differences, indicating the best treatment effect. In conclusion, the treatment effect of blepharitis could be promoted with the improved watershed algorithm, and the microscopic images combined with meibomian gland microprobe gave the better effect in the treatment of demodectic blepharitis than the conventional drug heat compress.

## 1. Introduction

Demodectic blepharitis is a chronic inflammatory disease caused by demodex infection of the eyelid margin, infectious in a certain degree. It is rare in clinical practice and is easily ignored. In particular, when accompanied by epidemic keratoconjunctivitis lesions, it is easy to be diagnosed as viral keratitis [1]. It has been found that the detection rate of eyelash follicle demodex gradually increased with age; the detection rate was 13% of those 3-15 years old, 34% of those 19-25 years old, 69% of those 31-50 years old, 87% of those 51-70 years old, and 95% of those 71-96 years old. In patients with blepharitis, the infection rate of demodex also increased significantly. Demodectic blepharitis can be divided into the anterior blepharitis, posterior blepharitis, and holo-eyelid blepharitis, according to the types of demodex infection and the site of inflammatory reaction [2]. Its pathogenesis is not clear and may be related to the involvement of various factors, such as immune response, direct destruction, physical damage, and secondary pathogenic microorganism infection. Dead demodex in eyelash sacs and glands will also increase bacterial antigen release, which in turn leads to an inflammatory response in the body [3, 4]. The main clinical symptoms of blepharitis include eyelid margin congestion, dry eyes, foreign body sensation, photophobia, eye itching, and increased secretions. The most typical symptoms include cuff-like secretions at the root of the eyelashes; in severe cases, repeated madarosis may occur [5, 6]. The treatment of demodectic blepharitis is still mainly on the bases of physical methods such as heat compress and eyelid margin cleaning, as well as topical application of tea tree oil, metronidazole, and other drugs. But there is not a unified standard for related drug treatment. Etiological examination is the key to diagnosing demodectic blepharitis. The eyelashes are taken to microscopically examine the roots of eyelashes, which is the most simple and effective clinical method [7, 8]. With a common optical microscope examination, demodex mites in each stage can be observed. In vivo corneal laser confocal microscopy can be utilized for noninvasive real-time observation, and the changes of tissue cells can be directly observed from the cellular level. Multiple follicles can also be quickly detected, which has a higher detection rate. Patients with eyelash loss can still be examined in a noninvasive and painless manner. For patients with recurrent and refractory meibomian gland cysts, pathological examination can be performed [9, 10].

The article "Improved Watershed Algorithm-Based Microscopic Images Combined with Meibomian Gland Microprobe in the Treatment of Demodectic Blepharitis" was published in 2022. Journal: Comput Math Methods Med.

Machine learning under computer intelligence makes it easier to identify and analyze data. Traditional classification processors are on the basis of manual work, which is time-consuming with large errors and relatively low recognition accuracy, so it cannot present image quality well [11–13]. The watershed algorithm is a mathematical morphology segmentation method under topology theory, which is fast in operation and accurate in positioning. For the grayscale value of each pixel in the image, the concept and formation of the watershed can be illustrated by the simulating intrusive process [14, 15]. The watershed algorithm consists of the intrusive watershed algorithm and the precipitation watershed algorithm. A fast algorithm under the precipitation watershed has been proposed in some works. Compared with the traditional algorithm, the algorithm is more sensitive to the edge and is prone to oversegmentation and undersegmentation [16, 17]. Label extraction in the image is a method of controlling oversegmentation. The above labels are used to compulsorily modify the minimum value region of the original gradient image, and the irrelevant minimum values in the original gradient image are masked. Thus, compared with the watershed method, it has a greater segmentation effect [18].

This research was to overcome the oversegmentation in the watershed algorithm, ensure the authenticity of microscopic image segmentation, and avoid distortion in image segmentation. The watershed algorithm was applied to the processing network of microscopic images and then combined with the meibomian gland microprobe to explore its effect in the treatment of demodectic blepharitis. It was expected to offer some help for clinical diagnosis and treatment.

## 2. Methodology

### 2.1. Research Objects

Patients with demodectic blepharitis-related dry eyes were taken as the research objects, who were in hospital from January 2018 to January 2020. There were 90 cases who met the criteria, including 36 males and 54 females; the age ranged from 50 to 78 years old, with an average of 54.53 ± 4.72 years. In the experimental group 1 (group E1) (*n* = 30), the microscopic images under the watershed algorithm and the microprobe were applied to dredge the blocked meibomian gland ducts; then, drugs, heat compress, massage, and other treatments were given. In the experimental group 2 (group E2) (*n* = 30), the blocked meibomian gland ducts were dredged with only the microprobe, combined with drugs, heat compress, massage, and so on. In the control group (group CG) (*n* = 30), patients were treated with conventional drugs, heat compress, and meibomian massage. The breakup time (BUT) of the tear film and the number of mites before and after treatment were compared among the three groups. There was no significant difference in the gender ratio and average age of the patients (*P* > 0.05). This research had been approved by ethics committee of hospital, and all patients and their families got to know and signed the informed consent form.

The article "Improved Watershed Algorithm-Based Microscopic Images Combined with Meibomian Gland Microprobe in the Treatment of Demodectic Blepharitis" was published in 2022. Journal: Comput Math Methods Med.

Inclusion criteria were as follows: the patients were in line with both the 2013 expert consensus on clinical diagnosis and treatment of dry eye disease and the Chinese expert consensus on the diagnosis and treatment of demodectic blepharitis (2018), and they were included in this experiment. They join this research voluntarily. They had no mental disorders, consciousness disturbances, and sleep disturbances.

Exclusion criteria were as follows: the patients who had non-demodex-infected blepharitis and who had dry eyes after eye surgery were excluded. Patients cannot take care of themselves with slurred speech, serious illness, etc. so that they cannot cooperate with the survey, or patients did not agree to participate in the research. Patients wore orthokeratologic lenses for a long term and had dry eye disease due to indiscriminate use of eye drops.

### 2.2. Meibomian Gland Microprobe

The meibomian gland microprobe was made of the national standard no. 7 metal injection needle. The needle tip and part of the needle tube were cut off, and the national standard 0.16 mm × 35 mm acupuncture needle was inserted into the needle tube until the needle tube was pierced. The main body of the probe was exposed with 4.5 mm. The needle exposed was broke over at 75°C; then, meibomian gland microprobe I was prepared already. Probe II was selected to expand the central gland duct. The needle core was a national standard 0.2 *μ*m × 35 *μ*m acupuncture needle, and the probe was connected to a 1 mL injection syringe.

### 2.3. The Watershed Algorithm

When utilizing the marked watershed algorithm, the minimum was forced to mark the algorithm. The minimum value region in the image was defined, and the extracted marker was forced to be the minimum value of the gradient image. Then, the watershed algorithm was applied. Inner and outer markings could be used to segment the region of interest. Inner marking was for the segmentations made for regions of minimum value. The outer marking used the watershed as an outer marker, and thresholding could be utilized to separate the background and the target of the segmented region. The watershed algorithm was an iterative labeling process, and the watershed mainly included sorting and submerging processes. The schematic diagram of this algorithm is displayed in Figure 1.

The specific mathematical process was described as follows.

If the function *g* on *W*_*g*_ in the definition domain was the image to be processed, the maximum and minimum values were expressed, respectively, as

(1) $$\begin{array}{c} {\text{h}}_{\max}=\max\left(g\right), \end{array}$$

(2) $$\begin{array}{c} {\text{h}}_{\min}=\min\left(g\right). \end{array}$$

The set [*W*_*g*_]*h* was the upper threshold of the function *g*; then, equations (3), (4), and (5) were worked out.

(3) $$\begin{array}{c} \left[{\text{W}}_{\min}\right]\text{h}=\left\{x\subseteq W_{g}\left|g\left(x\right)\right.\leq h\right\}, \end{array}$$

(4) Reg‐Minkg=x⊆Wgx=Local minimum,

(5) $$\begin{array}{c} g\left(x\right)=h. \end{array}$$

*X*_*h*max_ and *X*_*h*min_ were selected to represent the sets in the watershed region. Equation (6) was obtained after iteration.

(6) Xhmin=Whmin,Xhmin=Reg−Minh+1Ff∪IZWhminXh,∀h∈hmin,hmax−1.

The article "Improved Watershed Algorithm-Based Microscopic Images Combined with Meibomian Gland Microprobe in the Treatment of Demodectic Blepharitis" was published in 2022. Journal: Comput Math Methods Med.

During the rising of the water surface, the dam between the catchment basins would record the process of the skeleton point of the geodesic influence region of *X*_*h*max_.

The extended minimum transformation operation was the extreme value marked on the gradient image, which limited the number of local minimum points. When the depth threshold *W* was set, the local minima in the catchment basins below a given threshold were eliminated. The gradient image Δ*Q* was subjected to the depth threshold-extension minimum transformation operation, and the expression was

(7) $$\begin{array}{c} \Delta Q^{\text{Mark}}=\text{Wmin}\left(\Delta Q\;\left|\text{W}\right.\right). \end{array}$$

In the equation, Δ*Q*^Mark^ represented the marked gradient image, Δ*Q* represented the filtered gradient image, and *W*_min_ represented the minimal transformation in the morphological extension. After the gradient image was marked by the extreme value, the marked image was corrected by forced minimum operation. The local minimum region of the image appeared at the marked position, and the corrected image was corrected again using

(8) $$\begin{array}{c} \Delta Q=\text{IF}\min\left(\Delta Q\left|\Delta Q^{\text{mark}}\right.\right). \end{array}$$

In equation (8), IFmin stood for the morphological minimum value calibration operation.

### 2.4. The Improved Watershed Image Segmentation (IWS) Algorithm

In the watershed algorithm, the Sobel operator was used for edge extraction at first and then converted into gradients. In the process of image segmentation, it was easy to cause unclear image segmentation effect. The image segmentation algorithm under spatial pattern clustering was proposed to combine with the watershed. The image was segmented by the watershed algorithm, and then, the characteristic quantity of each watershed was defined. According to the different characteristic quantities, the spatial distance and Euclidean distance between similar regions were calculated. Finally, the distance of the pixel clustering center was determined (Figure 2).

The image segmentation algorithm was applied to the clustering algorithm. The fuzzy *C*-means (FCM) clustering technology was a clustering algorithm that determined the degree of each point belonging to a certain cluster by the degree of membership. This algorithm was used for merging the similar small regions generated by the watershed algorithm.

The article "Improved Watershed Algorithm-Based Microscopic Images Combined with Meibomian Gland Microprobe in the Treatment of Demodectic Blepharitis" was published in 2022. Journal: Comput Math Methods Med.

*D*_*i*_ was defined as the *i*-th region, and the clustering of the clustering center *V*_*i*_ and the pixel *X*_*k*_ was expressed as

(9) $$\begin{array}{c} \text{d}\left(x_{k},v_{i}\right)={\left(\frac{d_{ik}^{E}}{R+D_{ik}^{S}}\right)}^{2}. \end{array}$$

*D*_*ik*_^*S*^ was the spatial distance between the pixel and the cluster, while *d*_*ik*_^*E*^ was the Euclidean distance between the pixel and the cluster. *R* was the grayscale with a value of 256. The membership degree of adjacent domain pixels was mainly determined by the spatial distance. In this research, the membership degree of each pixel clustering center was determined, and the spatial distance was expressed as

(10) $$\begin{array}{c} d_{ik}^{s}=1-\frac{\sum_{l\in \eta s}\mu_{rt}\beta_{t}}{\sum_{c=1}^{c}\sum_{l\in \eta s}\mu_{rt}\beta_{t}}. \end{array}$$

0 ≤ *μ*_*rt*_ ≤ 1, and *μ*_*rt*_ was the membership degree of the pixel *S* belonging to the *r*-th cluster *V*_*r*_. *β* was the contribution factor of the neighborhood pixels, and *c* was the expected number of clusters.

With equation (9), the objective function of the clustering method under the spatial pattern was expressed as

(11) $$\begin{array}{c} {}_{7}Q_{m}\left(U,V\right)=\overset{n}{\underset{k=1}{\sum }}\overset{c}{\underset{i=1}{\sum }}{\mu^{\text{m}}}_{ik}d^{2}\left(x_{k},v_{i}\right), \end{array}$$

(12) $$\begin{array}{c} \overset{c}{\underset{k=1}{\sum }}\mu_{ik}=1,\;1\leq k\leq n. \end{array}$$

The membership function derived from the distance feature was

(13) $$\begin{array}{c} \mu_{ik}=\frac{{\left[d\left(x_{k},v_{i}\right)\right]}^{-2/\left(m-1\right)}}{\sum_{j=1}^{c}{\left[d\left(x_{k},v_{i}\right)\right]}^{-2/\left(m-1\right)}}. \end{array}$$

The specific flow of the IWS algorithm is shown in Figure 3.

The experimental environment adopted MATLAB 6.5. The experimental images were in the size of 256 × 256, the number of clusters was 2, and the grayscale was 256. The computer graphics card used was Intel 82865G, PC P4T23101.86G, 2 G RAM. 100 images were chosen for the training of the IWS algorithm.

### 2.5. Collection of Microscopic Images

The patients experienced slit-lamp examination and fundus examination for 3 times to exclude inner eye diseases, and then, the etiology of the eyelid was examined. Demodex mites were counted under the microscope. The eyes with severe clinical symptoms were selected, and 5 eyelashes were extracted with sterile tweezers and placed on a glass slide with 10% potassium hydroxide. The eyelashes with sleeved secretions at the root were selected as possible. Cedar oil was added dropwise; 5 minutes later, a cover glass was covered. They were observed under a 30x optical microscope to count the number of demodex mites.

The article "Improved Watershed Algorithm-Based Microscopic Images Combined with Meibomian Gland Microprobe in the Treatment of Demodectic Blepharitis" was published in 2022. Journal: Comput Math Methods Med.

### 2.6. Evaluation Indicators for the Treatment Effect

For subjective clinical symptoms, the scale included 8 items including dry eyes, blepharitis, photophobia, eye itching, eye burning sensation, foreign body sensation, increased secretion, and eyelash loss. Then, the scale was scored according to the duration and severity of symptoms. The sum of the scores for 8 items ranged from 0 to 24; the higher the score, the more severe the symptoms. The persistence of symptoms that seriously affected life was scored as 3 points, most of the symptoms occurring with the moderate discomfort were scored as 2 points, the occasional symptoms not affecting daily life was scored as 1 point, and no symptom was scored as 0 point.

The clinical sign score included that of conjunctival hyperemia, meibomian gland secretion characteristics, meibomian gland opening blockage, and microscopic examination of phosphorous debris at the root of the eyelashes. The total score of the 4 signs was 12 points; the higher the score, the more serious the condition (Table 1).

Treatment effect criteria were described as follows. The subjective symptoms disappeared, meibomian gland opening was unobstructed, no foreign body secretion was extruded, and BUT of the tear film was normal or close to normal (≥8 s); these were regarded to be self-cured. Subjective symptoms were significantly relieved, most of the meibomian gland opening was unobstructed, no or slight abnormal secretions overflowed during extrusion, and the BUT of the tear film was much longer than before (the extension ≥ 3 s). These were regarded as effective. Most of the opening of the meibomian gland was obstructed, the subjective symptoms were not improved obviously, the abnormal secretions still overflowed, and the BUT of the tear film did not change markedly; thus, the treatment was ineffective.

The average noninvasive keratography break-up time (NIKBUTav) was checked in a dark room, using the comprehensive treatment device Keratograph 5M. The patients were instructed to sit in the correct posture, facing the instrument in front. After the infrared light was turned on, the patients blinked twice for the examinations. Then, the patients should keep the eyes open until the BUT of the tear film was recorded by the system. The NIKBUTav was obtained as the average was calculated from the results of three times.

The article "Improved Watershed Algorithm-Based Microscopic Images Combined with Meibomian Gland Microprobe in the Treatment of Demodectic Blepharitis" was published in 2022. Journal: Comput Math Methods Med.

### 2.7. Statistical Methods

SPSS21.0 software was applied for statistical analysis of the parameters to be analyzed. The measurement data conforming to the normal distribution were expressed as mean ± standard deviation ($\bar{x}\pm s$), and the nonconforming enumeration data were expressed as frequency (%). *α* = 0.05 was taken as the test standard for comparison between groups. When *P* < 0.05, the difference was considered to be statistically significant.

## 3. Results

### 3.1. Analysis of the Algorithm

The improved algorithm in this work was compared with the algorithms researched by other scholars, as shown in Figure 4. The *F*-measure value of the IWS algorithm proposed here was superior to that of other segmentation algorithms. Compact watershed segmentation (CWS) [19], Normalized Cut (NCUT) [20], and Mean Shift (MSHIFT) [21] algorithms still had much room for the improvement in the *F*-measure.

### 3.2. Treatment for Patients

The general data of the three groups of patients were analyzed and compared, as shown in Table 2. The results indicated that there was no significant difference among the three groups (*P* > 0.05).

### 3.3. Images of Demodex Mites

Figure 5(a) represents a shield-shaped or irregular oval-shaped mite (400x), and Figure 5(b) shows that the larvae had constricted on the side of the body (400x). In Figure 5(c), the body of the demodex mite was thinner and had differentiated into 4 pairs of legs (400x). The size of the adult mite in Figure 5(d) was 0.17-0.44 mm (400x).

### 3.4. Microscopic Images of Demodex Mites

Figure 6(a) shows the eyelid margin with eyelashes. Demodex mites could be observed in the hair shaft of the eyelashes in Figure 6(b).  Figure 6(c) is a microscopic image, and in Figure 6(d), there were 3 adults and 1 egg of the demodex mites on the surface of the root of the eyelashes (the position marked by the red dotted box).  Figure 6(f) presents that the demodex mites were observed on the hair shaft of the eyelashes after being wiped with drugs. The clear image after algorithm processing was obtained as Figure 6(e).

### 3.5. Structural Comparison of BUT before and after Treatment in Three Groups

The NIKBUTav of patients in the three groups was analyzed and compared. The effects of both group E1 and group E2 after treatment were significantly better than those before treatment, with the significant differences (*P* < 0.05). No significant difference was obtained in the NIKBUTav before and after treatment (*P* > 0.05) (Figure 7).

### 3.6. Comparison of Clinical Symptom Scores of Patients in Three Groups before and after Treatment

As shown in Table 3, there was a significant difference between group E1 and group E2 compared with the scores before treatment (*P* < 0.05). For the score of subjective clinical symptoms in group E1, the difference was the largest before and after treatment; thus, the treatment effect was the best.

The article "Improved Watershed Algorithm-Based Microscopic Images Combined with Meibomian Gland Microprobe in the Treatment of Demodectic Blepharitis" was published in 2022. Journal: Comput Math Methods Med.

As shown in Table 4, the scores of clinical signs in group E1 and group E2 after treatment were significantly different from those before treatment (*P* < 0.05). There was the biggest difference in group E1, showing the best treatment effect.

### 3.7. Comparison of the Number of Demodex Mites in the Three Groups before and after Treatment

There was no significant difference in the number of demodex mites among the three groups before treatment (*P* > 0.05). No significant difference was also found in the number of demodex mites in the CG group before and after treatment (*P* > 0.05). After treatment, the number of demodex mites in group E1 and group E2 was highly reduced than that before treatment, and the difference was of statistical significance (*P* < 0.05) (Figure 8).

## 4. Discussion

Blepharitis will occur in all-age population. Meibomian gland opening, the most important structure of the eyelid margin, is easily invaded by blepharitis. Meibomian gland probing is a recognized and effective method in the treatment of meibomian dysfunction and meibomian gland obstruction. The meibomian gland microprobe can be used to dredge the meibomian gland duct with a good effect on the treatment of meibomian gland dysfunction. Patients with meibomian gland dysfunction have increased free fatty acids, which forms foam image affecting tear film stability, and elevated cholesterol causes dry eye syndrome [22, 23]. Randon et al. [24] illustrated that in vivo confocal microscopy could identify demodex mites, and focusing microscopy was an effective and reliable diagnostic tool. This research also showed that microscopy could be utilized for the diagnostic identification of demodex mites. In this work, the microscopic images were combined with the meibomian gland microprobe, and the watershed algorithm was introduced into the microscopic images for image segmentation and denoising. The treatment effect of group E1 was remarkably better than that of the other two groups (*P* < 0.05). The topical physical nursing in this research included eyelid margin cleaning, eye massage, and eye heat compress. Eyelid margin cleaning was mainly to use cotton swabs dipped in sterile saline or use eye cleaning wipes to clean the roots of eyelashes, so as to remove scales and scabs on eyelid margins. Eye massage was to help remove the secretions that blocked meibomian glands. Eye heat compress was to soften the lipids in the meibomian and sebaceous glands, accelerating the excretion of meibomian lipids. For patients with severe blepharitis reaction during treatment, local administration of glucocorticoid eye ointment could effectively reduce the blepharitis reaction. For patients with keratoconjunctival lesions, the low-concentration glucocorticoid eye drops were given to relieve inflammatory reactions obviously. After the ocular reaction control, the treatment was maintained with less irritating anti-inflammatory drugs.

The article "Improved Watershed Algorithm-Based Microscopic Images Combined with Meibomian Gland Microprobe in the Treatment of Demodectic Blepharitis" was published in 2022. Journal: Comput Math Methods Med.

At the current stage, segmentation algorithms in computer vision get applications in the segmentation of image characteristics, but there is no sign for evaluating the quality of the algorithms. The watershed algorithm has been mainly researched focusing on reducing the oversegmentation during the growth process. In the process of reducing the sensitivity of the watershed to noise data, the oversegmentation can be solved, but how to optimize the gradient information is also very important [25, 26]. Bonanno et al. [27] used a hybrid watershed clustering algorithm for the diagnosis of multiple sclerosis lesions, which could distinguish lesions from nonlesions. The proposed method produced detections that could support clinical evaluation. In this research, watershed and clustering algorithms were utilized for processing the microscopic images of demodectic blepharitis. With good results, the algorithm system server processed 4,887 data per minute, and the success rate was about 96.2%. The concurrency of the system platform could basically meet the requirements and satisfy the needs of users. This suggested that the algorithm could be used for the evaluation of clinical eyelid diseases. The watershed algorithm was combined with clustering technology and then applied to the image denoising and segmentation. The watershed algorithm performed boundary extraction on the clustered target data. Compared with that, the segmentation regions were obtained by clustered data via binarization, the edges here were clearer and neater, and the dividing line was more precise and reliable.

## 5. Conclusion

In this work, the watershed algorithm was applied to the treatment of demodectic blepharitis combining with microscopic images as well as meibomian gland microprobes. The IWS algorithm had a great segmentation effect in the feature segmentation and extraction of images and could reduce the oversegmentation of watershed. Meibomian gland microprobe had a certain effect in the treatment of demodectic blepharitis. The IWS algorithm under the watershed algorithm had a good application prospect in treating demodectic blepharitis; it was safe and reliable and was worthy of clinical promotion. Although the IWS algorithm could have a good segmentation effect, in the experimental process, whether the automatic selection of parameters could be realized in combination with the theory needed to be further discussed. The samples in this work were limited, and more samples were needed to further research the evaluation of the treatment effect.

The article "Improved Watershed Algorithm-Based Microscopic Images Combined with Meibomian Gland Microprobe in the Treatment of Demodectic Blepharitis" was published in 2022. Journal: Comput Math Methods Med.

## Figures and Tables

**Figure 1:** Schematic diagram of the watershed algorithm.

**Figure 2:** Image segmentation flowchart of the watershed algorithm.

**Figure 3:** The specific flowchart of the IWS algorithm.

**Figure 4:** Analysis results of different algorithms.

**Figure 5:** Images of demodex mites.

**Figure 6:** Microscopic images of demodex mites.

**Figure 7:** Comparison of NIKBUTav of patients among the three groups before and after treatment. ^∗^Compared with that before treatment (*P* < 0.05).

**Figure 8:** Comparison of the number of demodex mites in the three groups before and after treatment. ^∗^Compared with those before treatment (*P* < 0.05); ^#^compared with CG (*P* < 0.05).

**Table 1:** The scoring scale of various symptoms.

Scoring items		Symptoms	Score
Subjective symptoms		Asymptomatic	0
		Occasionally, not affecting daily life	1
		Mostly, moderate discomfort	2
		Persistence of symptoms seriously affecting life	3
Sign score	Blockage of meibomian gland opening by phosphorous debris at the root of eyelashes	None	0
		<1/3 eyelid margin	1
	Meibomian gland secretion	Clear	0
		Dirty	1
		Granular or chyle	2
		Toothpaste-shaped	3
	Conjunctival hyperemia	None	0
		Mild	1
		Moderate	2
		Severe	3

**Table 2:** General information of patients.

Groups	Number	Man	Women	Average age
E1	30	11	19	51.06 ± 2.13
E2	30	13	17	49.60 ± 4.34
CG	30	20	10	
Total	90	44	46	53.56 ± 2.34

**Table 3:** Comparison of scores of subjective clinical symptoms of patients among the three groups.

Groups	Before treatment	After treatment	*t*	*P*
E1	13.43 ± 1.41	3.1 ± 1.841^∗^^#^	21.75	<0.001
E2	13.51 ± 1.41	5.4 ± 0.661^∗^	19.272	<0.001
CG	13.64 ± 0.84	13.4 ± 0.841	1.432	0.142
*F*	0.026	587.32		
*P*	0.875	<0.001		

^∗^Compared with those before treatment (*P* < 0.05); ^#^compared with those in group E2 (*P* < 0.05).

**Table 4:** Comparison of clinical sign scores of patients among the three groups.

Groups	Before treatment	After treatment	*t*	*P*
E1	7.23 ± 1.371	3.1 ± 1.841^∗^#	11.74	<0.001
E2	7.31 ± 1.414	5.4 ± 1.161^∗^	8.279	<0.001
CG	7.61 ± 0.93	6.75 ± 0.641	1.331	0.247
*F*	0.042	187.71		
*P*	0.893	<0.001		

^∗^Compared with those before treatment (*P* < 0.05); ^#^compared with CG (*P* < 0.05).

## Data Availability

The data used to support the findings of this study are available from the corresponding author upon request.
